RETRACTED

# Efficacy and Risk Factors of Pyrrotinib in Second- and Third-Line Treatments for HER2-Positive Advanced Breast Cancer

**DOI:** 10.1155/2022/7864114

**Published:** 2022-09-17

**Authors:** Xiaolei Wang, Yuxia Huang, Zhen Yang, Yang Yang, Fenfen Wei, Min Yan, Fanfan Li

**Affiliations:** ^1^Department of Oncology, The Second Affiliated Hospital of Anhui Medical University, Hefei 230601, China; ^2^Department of Medical Oncology, Chizhou Second People's Hospital, Chizhou, Anhui 247100, China

## Abstract

A study to examine the efficacy and risk factors associated with pyrrotinib in the second- and third-line treatment of advanced breast cancer with Human epidermal growth factor receptor 2- (HER2-) positive cells was conducted. Progression-free survival (PFS) was assessed as the primary endpoint, and the objective response rate (ORR), overall survival (OS), and safety were secondary endpoints. Across all the patients, the ORR was 48.57%, and the disease control rate (DCR) was 94.29%. In the follow-up period, the median PFS was 15 months, and second-line treatment had significantly longer PFS than third-line treatment (*P* = 0.027). The OS among all the patients was up to 28 months, but the median OS has not yet been reached. Diarrhea (69.57%) was the most important AE, mainly in grades 1 and 2. According to the COX regression analysis, brain metastasis was a risk factor for PFS, while second-line treatment and capecitabine chemotherapy were relevant to a longer PFS correlation among patients. In the second- and third-line treatment, pyrrotinib is still highly effective and safe. Pyrrotinib is a potential ideal salvage treatment plan for patients who failed in first-line treatments.

## 1. Introduction

Breast cancer, the leading cause of cancer death in women, is the most common malignant cancer in women [1, 2]. The latest data on the global cancer burden showed more than 2.26 million new cases of breast cancer and 2.2 million lung cancer in 2016, and breast cancer became the most prevalent cancer in the world [3, 4]. Breast cancer is a highly heterogeneous tumor with diverse histological morphology and genotypes. Human epidermal growth factor receptor 2- (HER2-) positive breast cancer refers to ERBB2/neu protooncogene amplification or HER2 transmembrane receptor protein overexpression, which accounts for about 15%–20% of all breast cancers in incidence [5, 6]. HER2-positive breast cancer is characterized by its proclivity for recurrence, highly aggressive metastasis, rapid progression, and poor prognoses [7, 8]. Based on the characteristics, anti-HER2-targeted drug therapy is considered effective in inhibiting tumor progression and prolonging the survival of patients.

RETRACTED

With the continuous research into breast cancer's immune phenotype, more targeted drugs have been developed. Currently, the common clinical targeted therapy drugs for HER2-positive breast cancer mainly include tyrosine kinase inhibitors, monoclonal antibodies, and antibody-drug conjugates. However, the effect of targeted therapy in some patients has been unsatisfactory because of drug resistance. Therefore, it is necessary to develop more types of anti-HER2-targeted drugs. A new type of oral pan-ErbB receptor tyrosine kinase inhibitor, pyrrotinib, has been developed by China independently [9]. Its mechanism of action is as follows: it irreversibly binds to the ATP binding site of EGFR/HER1, HER2, and HER4 to prevent the formation of homo/heterodimers between the HER family, inhibit autophosphorylation, and block downstream signal transmission, thereby inhibiting tumor growth [9–11]. The actual effect of pyrrotinib in clinical application still needs more case support, even though it has achieved high evaluations in clinical trials I, II, and III phases [12, 13]. The effectiveness in treating HER2-positive breast cancer in first-line treatment has been proved, while no reports have explored the efficacy in second-line and third-line treatment. What is important is that previous studies were limited to the analysis of treatment effects and ignored the observation of factors affecting treatment efficacy.

We review the efficacy of pyrrotinib in the second- and third-line breast cancers with HER2-positive and analyze the factors that affect treatment efficacy in this study. This is the first evidence-based study to analyze the factors affecting the efficacy of pyrrotinib in HER2-positive breast cancer.

## 2. Methods

### 2.1. Patient

Thirty-five patients with HER2-positive breast cancer treated with pyrrotinib between December 2018 and October 2021 were admitted to the study. Clinical data were complete in all patients. Inclusion criteria are as follows: (1) patients met the diagnostic criteria for HER2-positive breast cancer; that is, their primary or metastatic tissue specimens were immunohistochemically HER2 positive (“+++”) or exhibited positive fluorescence in situ hybridization (FISH) (“+”); (2) patients were adult females; (3) patients had at least one measurable lesion, meeting the curative effect according to the response evaluation criteria in solid tumors (RECIST 1.1) evaluation conditions; (4) the patients received pyrrotinib treatment regimens; (5) their expected survival time was at least three months; and (6) the patients' physical functions tolerated pyrrotinib treatment, and there were no treatment contraindications. Exclusion criteria are as follows: (1) patients were undergoing other clinical trials; (2) they lacked follow-up data; and (3) psychiatric patients who cannot receive medication.

RETRACTED

### 2.2. Ethical Statement

Based on meeting the Declaration of Helsinki, The Second Affiliated Hospital of Anhui Medical University (PY-YX2021-46) ethics committee approved this study. Studying retrospectively waived informed consent due to its retrospective nature.

### 2.3. Treatment Plan and Follow-Up

All patients received pyrrotinib for second-line or third-line treatment after the first-line. The patients took pyrrotinib maleate tablets orally (Jiangsu Hengrui Pharmaceutical Co., Ltd., National Medicine Zhunzi H20180013, 80 mg/tablet) at 4 tablets/320 mg, QD. After patients tolerated this regimen, the dose was increased to 5 tablets/400 mg, QD. Patients undergoing anti-HER2 second-line and third-line treatments were treated with combined chemotherapy regimens: capecitabine, tigeo, gemcitabine, taxanes, vinorelbine, and etoposide. Treatment efficacy was evaluated every two cycles (every six weeks). Treatment plans were adjusted when patients had grade 1 (mild reactions, no treatment required) or 2 (moderate response, requiring treatment) side effects. When side effects of grade 3 (severe reaction, life-threatening but recoverable) and above occurred, the dosages of the drugs were adjusted according to the types of side effects, or the number of combined chemotherapy drugs was reduced. All patients received long-term follow-ups, and the end of their follow-up period was defined as disease progression or the intolerance of treatment. All patients completed the study, and no patients dropped out of the study halfway through.

### 2.4. Treatment Efficacy and Adverse Events (AEs) Evaluation

Based on the RECIST (version 1.1), efficacy was evaluated [10] as complete response (CR), partial response (PR), stable disease (SD), and disease progression (PD). The objective response rate (ORR) is the sum of the proportions of CR and PR, and the disease control rate (DCR) is the proportions of CR, PR, and SD. In addition, all patients' survival times were recorded in detail.

AEs were classified into grades 1 through 5 based on National Cancer Institute Common Terminology Criteria for Adverse Events (NCI-CTC 4.0) [11].

### 2.5. Risk Factor Analysis Strategy

To analyze risk factors, ORR and PFS, AEs grade 3 or higher were used as dependent variables. Age, ECOG scores, WHO grades, ER, PR, P53/P63, pathological type, comorbidities, surgery, vascular tumor thrombus, the combined chemotherapy regimen, the number of pyrrotinib treatment lines, and the location of metastasis were used as dependent variables. The single-factor and multifactor logistic regression or the COX regression analysis models were used for correlation analysis.

RETRACTED

### 2.6. Statistical Analysis

We performed statistical analysis by SPSS 26.0. We expressed enumeration data as cases (percentage) [*n* (%)], and performed the *χ*^2^ test to test for significance. We analyzed correlations via the single-factor and multifactor logistic regression or the COX regression analysis models. The Kaplan-Meier survival curve was used to evaluate the survival time of patients. *P* < 0.05 means the difference was significant.

## 3. Results

### 3.1. Baseline

35 breast cancer patients with HER2-positive were included, including 22 second-line cases and 13 third-line cases involving pyrrotinib. The patients aged 29 to 70 years (average of 49.4 ± 9.3 years). In addition, 71.43% of the patients had an ECOG score less than or equal to 1 at the start of treatment. Most patients (62.86%) had a WHO classification of grade 2, and only two patients had a family history of breast cancer. The main combination chemotherapy regimen was capecitabine (40.00%), followed by albumin paclitaxel (22.86%).  Figure 1 shows the details of pyrrotinib use, and there were no statistical differences in baseline data between the groups (*P* > 0.05) (Table 1).

### 3.2. The Efficacy of Pyrrotinib

Table 2 shows the best response to pyrrotinib targeted therapy for all HER2-positive breast cancer patients which can be assessed. Only two patients achieved CR (1 in second-line and 1 in third-line treatment), and 15 patients achieved PR (12 in second-line and 3 in third-line treatment). A total of 15 cases reached SD, and 3 cases with PD. The ORR was 48.57%, and the DCR was 94.29%. There was no significant difference in ORR and DCR between second-line and third-line treatment (*P* > 0.05) regimens. As the follow-up period ended, 26 patients (17 in the second-line and 9 in the third-line) survived, with a survival rate of 74.29%.

As of follow-ups to December 2021, 16 patients had progressed (8 in second-line and 8 in the third-line treatment). Their PFS was as high as 28 months, and the median PFS was 15 months (Figure 2(a)). PFS was significantly longer than in third-line treatment (HR = 0.27, 95% CI: 0.087–0.862, *P* = 0.027) (Figure 2(b)).

At the end of the follow-up period, 26 patients (74.29%) were alive; seven had passed away, and two were lost to follow-up. The overall OS was 2–28 months, but the median OS was not yet reached (Figure 1(a)). No significant difference was observed in OS between second-line and third-line treatment patients (HR = 1.16, 95% CI: 0218–06.158, *P* = 0.864) (Figure 1(b)).

### 3.3. Safety Analysis of Pyrrotinib

AE details are shown in Table 3. The most common side effect of the patients in the study was diarrhea, with an incidence of 69.57%, but grade 3 diarrhea was rare, with only three cases that have occurred. Diarrhea was relieved after reducing drug dosages until it was reduced to grade 1. Five patients had grade 2–3 neutropenia, and one case of grade 3 thrombocytopenia was documented. Other side effects were observable, including anemia, vomiting, skin rashes, hand-foot syndrome, elevated transaminase, hypertension, and peripheral neuritis. Their incidence was low, and there were no grade 3 AEs.

RETRACTED

### 3.4. Risk Factors for the Efficacy of Pyrrotinib

We further incorporated the significant factors (*P* < 0.01) into a multivariate logistic regression model. The analysis results showed that after excluding confounding factors, comorbidities (OR = 1.380, 95% CI: 1.027–1.664) were independent factors influencing the ORR of pyrrotinib during the treatment. In addition, surgery (OR = 0.905, 95% CI: 0.695–0.980) was associated with a higher ORR (Table 4).

In the univariate analysis, variables related to PFS were obtained, including age, ECOG score, the number of treatment lines, pyridoxine chemotherapy drugs, pathological types, and brain metastases. After incorporating them into a multivariate model for further analysis, the results showed that after controlling for other potential confounding factors, brain metastasis (HR = 1.425, 95% CI: 1.138–2.502) was an independent risk factor for PFS, while second-line treatment (HR = 0.362) and capecitabine chemotherapy (HR = 0.880) were associated with a longer PFS (*P* < 0.05) (Table 5).

### 3.5. Risk Factors for the Safety of Pyrrotinib

Next, we analyzed the risk factors for the safety of pyrrotinib. Multivariate logistic regression analysis showed that patients 50 years old or older (OR = 1.263) and those with an ECOG score of 2 (OR = 1.185) were associated with more grade 3 AEs, whereas combined capecitabine chemotherapy (OR = 0.893) was associated with a reduced incidence of grade 3 AEs (Table 6).

## 4. Discussion

Pyrrotinib has been approved for HER2-positive advanced breast cancer treatment because of the significant outcomes in the recent phase II and phase III clinical studies in China [14, 15]. Previous studies, however, mainly analyzed the results of pyrrotinib applied to first-line treatment. Therefore, we focused on the efficacy and safety of pyrrotinib in second-line and third-line HER2-positive advanced breast cancer in this study, and by analyzing the treatment data of each patient, we sought to shed light on these issues.

This study showed that pyrrotinib is still significantly affected during the second-line and third-line treatment of HER2-positive advanced breast cancer. The overall ORR of the patients was as high as 48.57% (59.09% in the second-line treatment regimen and 30.77% in the third-line treatment regimen), and the DCR was as high as 94.29%. Although this ORR was not as ideal as the results of Phase II and III clinical studies [13, 16], considering the baseline characteristics of these local patients, the complexity of their combined chemotherapy regimens and the impact of the failure of patients' first-line treatments, these results were ideal. In addition, efficacy was improved compared with the currently recommended lapatinib [17, 18] combined chemotherapy regimen (48.57% vs. 34.4%). In terms of survival, this cohort showed satisfactory PFS and OS. PFS was up to 28 months, the median PFS was 15 months, and OS was up to 28 months. The median OS has not yet been reached. The median is predicted based on the survival curve. OS will reach 35 months.

RETRACTED

The NCCN guidelines list several treatment options for HER2-positive advanced breast cancer patients whose first-line treatment with trastuzumab failed [19–21]. These options include switching to a regimen containing lapatinib, continuous administration of trastuzumab while switching to other chemotherapeutic drugs, terminating chemotherapy, and trastuzumab plus lapatinib dual-targeted therapy and TDM1 administration. TDM1 is not yet available in China, and most patients are not suited for dual-targeted therapy. Also, patients often cannot afford the expensive anti-HER2 costs. As an anti-HER2-targeted drug independently developed by China, pyrrotinib has cost advantages, and more importantly, it seems to have a better effect in patients [22–24]. Most cases (27 cases) in this cohort were patients who failed first-line trastuzumab treatment. After pyrrotinib was combined with chemotherapy, 94.29% (33 cases) of the patients showed clinical improvement and had survived by the end of the follow-up period, with a rate as high as 74.29% (26 cases). Combined with the results of this study, we believe that for most Chinese patients with HER2-positive advanced breast cancer and who underwent failed first-line treatments with trastuzumab, pyrrotinib plus chemotherapy is most likely the new ideal choice.

The efficacy of pyrrotinib in the second-line and third-line treatment was observed. The ORR, DCR, and OS were not significantly different, while the median PFS of second-line treatment patients was higher than third-line. Treatment times were also significantly longer. This may have been due to the greater tolerance of targeted therapy and (or) chemotherapy drugs among third-line treatment patients after first-line and second-line treatment [25–27]. In addition, current studies rarely analyze the potential influencing factors of the efficacy of pyrrotinib. Therefore, we further analyzed the possible influencing factors of patients' ORR and PFS. The results showed that after excluding confounding factors, comorbidities (OR = 1.380, 95% CI: 1.027–1.664) were independent factors influencing the ORR of pyrrotinib during the treatment, and surgery was associated with a higher ORR. For PFS, brain metastasis (HR = 1.425), the number of medication lines (HR = 0.362), and capecitabine chemotherapy (HR = 0.880) are potential influencing factors identical to those of the previous trastuzumab treatment [28–31].

RETRACTED

Regarding safety, diarrhea was still the most common side effect among patients, but diarrhea above grade 3 was rare, consistent with the previous study. One patient developed grade 3 neutropenia and thrombocytopenia at the same time. This patient changed chemotherapeutic drugs twice in succession; thus, these side effects were considered to be caused by chemotherapeutic drugs. The incidence of other AEs was relatively low, especially for vomiting and hand-foot syndrome. Compared with lapatinib, pyrrotinib is an irreversible tyrosine kinase inhibitor whose mechanism of action is different [23]. Similarly, multivariate logistic regression analysis showed that an age of 50 years old or older (OR = 1.263) and an ECOG score of 2 (OR = 1.185) were associated with a greater incidence of grade 3 AEs. In contrast, combined capecitabine chemotherapy (OR = 0.893) was associated with a lower incidence of grade 3 AEs, suggesting that capecitabine can be selected as a combination chemotherapy regimen to reduce the occurrence of adverse reactions.

There are 2 limitations to this study. First, the small sample size and the lack of a single center limited the applicability of the research results. In addition, this study was a retrospective study without prospective randomization. Therefore, there may have been significant biases in the sociological characteristics, physiological status, tumor characteristics, and other baseline characteristics of the patients. There was a difference in the number of combined chemotherapy drugs between the two groups. Despite these limitations, this was the first observational study to analyze the use of pyrrotinib for the second-line and third-line treatment of HER2-positive advanced breast cancer. It initially demonstrates the use of pyrrotinib in such second-line and third-line treatment and the huge potential of its full-line treatment. Also, combined with an analysis of efficacy and factors influencing safety, this study can be a useful reference for clinical practice.

RETRACTED

## 5. Conclusion

Pyrrotinib combined with chemotherapy has good efficacy and high safety in the second- and third-line treatment of HER2-positive advanced breast cancer.

## Figures and Tables

**Figure 1:** The overall survival of the patients. (a) The Kaplan-Meier curve of OS in patients undergoing second-line and third-line treatment, where the log-rank *P* > 0.05 between groups; (b) the Kaplan-Meier curve of OS in all patients.

**Figure 2:** The progression-free survival of patients. (a) The Kaplan-Meier curve of PFS in patients undergoing second-line and third-line treatment, where the log-rank *P* = 0.027 between groups; (b) the Kaplan-Meier curve of PFS in all patients. PFS refers to progression-free survival.

**Table 1:** Baseline data of breast cancer patients with HER2-positive.

Items	Second-line (*n* = 22)	Third-line (*n* = 13)	Total (*n* = 35)
Age (years)	50.9 ± 9.5	46.5 ± 8.8	49.4 ± 9.3
ECOG score [*n* (%)]			
0~1	16 (72.73)	9 (69.23)	25 (71.43)
2	6 (27.27)	4 (30.77)	10 (28.57)
WHO grade [*n* (%)]			
II	15 (68.18)	7 (53.85)	22 (62.86)
III	7 (31.82)	6 (46.15)	13 (37.14)
ER [positive, *n* (%)]	11 (50.00)	6 (46.15)	17 (48.57)
PR [positive, *n* (%)]	13 (59.09)	7 (53.85)	20 (57.14)
P53/P63 [positive, *n* (%)]	9 (40.91)	4 (30.77)	13 (37.14)
Pathological type [*n* (%)]			
Invasive carcinoma	11 (50.00)	6 (46.15)	17 (48.57)
Invasive ductal carcinoma	6 (27.27)	3 (23.08)	9 (25.71)
Other	5 (22.73)	4 (30.77)	9 (25.71)
Family history [yes, *n* (%)]	1 (4.55)	1 (7.69)	2 (5.71)
Complications [yes, *n* (%)]	5 (22.73)	2 (15.38)	7 (20.00)
Surgery [yes, *n* (%)]	15 (68.18)	10 (76.92)	25 (71.43)
Vascular tumor thrombus [positive, *n* (%)]	8 (36.36)	2 (15.38)	10 (28.57)
Combination chemotherapy [*n* (%)]			
Capecitabine	10 (45.45)	4 (30.77)	14 (40.00)
Albumin paclitaxel	6 (27.27)	2 (15.38)	8 (22.86)
Gemcitabine	2 (9.09)	2 (15.38)	4 (11.43)
Other	4 (18.18)	5 (38.46)	9 (25.71)

**Table 2:** The best response to pyrrotinib targeted therapy for all HER2-positive breast cancer patients.

Efficacy	Second-line (*n* = 22)	Third-line (*n* = 13)	Total
CR	1 (4.55)	1 (7.69)	2 (5.71)
PR	12 (54.55)	3 (23.08)	15 (42.86)
SD	8 (36.36)	7 (53.85)	15 (42.86)
PD	1 (4.55)	2 (15.38)	3 (8.57)
ORR	13 (59.09)	4 (30.77)	17 (48.57)
DCR	21 (95.45)	11 (84.62)	33 (94.29)
Survival rate [*n* (%)]	17 (77.27)	9 (69.23)	26 (74.29)

**Table 3:** The AEs of HER2-positive breast cancer patients [*n* (%)].

AEs	Grade			Total
	1	2	≥3	
Hematological AEs				
Anemia	3	2	0	5
Neutropenia	0	2	3	5
Thrombocytopenia	0	0	1	1
Non-hematological AEs				
Diarrhea	19	3	3	25
Vomiting	1	0	0	1
Skin rash	2	0	0	2
Hand-foot syndrome	2	0	0	2
Other AEs				
Elevated transaminase	1	0	0	1
Hypertension	3	0	0	3
Peripheral neuritis	2	1	0	3

RETRACTED

**Table 4:** Multivariate logistic regression analysis of ORR.

Variables	OR	95% CI	*P*
Age (>50 years old vs. ≤50 years old)	1.063	0.859~1.303	0.296
Comorbidities (yes vs. no)	1.380	1.027~1.664	0.020
Surgery (yes vs. no)	0.905	0.695~0.980	0.032
Pathological type (invasive cancer vs. other)	1.125	0.730~1.308	0.296

**Table 5:** Multivariate logistic regression analysis of ORR.

Variables	HR	95% CI	*P*
Age (>50 years old *vs* ≤50 years old)	1.132	0.806~1.362	0.239
ECOG score (2 points vs. ≤1 point)	1.285	0.859~1.933	0.088
Number of treatment lines (second-line vs. third-line)	0.362	0.119~0.895	0.005
Chemotherapy drugs (capecitabine vs. others)	0.880	0.567~0.994	0.036
Hormone status (positive vs. negative)	0.925	0.445~1.369	0.167
Pathological type (invasive cancer vs. other)	1.125	0.859~1.492	0.265
Brain metastasis (yes vs. no)	1.425	1.138~2.502	0.007

**Table 6:** Multivariate logistic regression analysis of the safety of pyrrotinib for the treatment of HER2-positive breast cancer.

Variables	OR	95% CI	*P*
Age (>50 years old *vs.* ≤50 years old)	1.263	1.059~1.738	0.042
ECOG score (2 points vs. ≤1 point)	1.185	1.032~1.835	0.035
Comorbidities (yes vs. no)	1.180	0.927~1.625	0.094
Chemotherapy drugs (capecitabine vs. others)	0.893	0.627~0.964	0.014

## Data Availability

The datasets used and analyzed during the current study are available from the corresponding author upon reasonable request.
